# Air-stable superparamagnetic metal nanoparticles entrapped in graphene oxide matrix

**DOI:** 10.1038/ncomms12879

**Published:** 2016-09-15

**Authors:** Jiří Tuček, Zdeněk Sofer, Daniel Bouša, Martin Pumera, Kateřina Holá, Aneta Malá, Kateřina Poláková, Markéta Havrdová, Klára Čépe, Ondřej Tomanec, Radek Zbořil

**Affiliations:** 1 Department of Experimental Physics and Department of Physical Chemistry, Regional Centre of Advanced Technologies and Materials, Faculty of Science, Palacky University in Olomouc, Slechtitelu 27, 783 71 Olomouc, Czech Republic; 2 Department of Inorganic Chemistry, University of Chemistry and Technology Prague, Technická 5, 166 28 Prague 6, Czech Republic; 3 Division of Chemistry & Biological Chemistry, School of Physical and Mathematical Sciences, Nanyang Technological University, 637371 Singapore, Singapore; 4 Institute of Scientific Instruments, The Czech Academy of Sciences, Kralovopolska 147, 612 64 Brno, Czech Republic

## Abstract

Superparamagnetism is a phenomenon caused by quantum effects in magnetic nanomaterials. Zero-valent metals with diameters below 5 nm have been suggested as superior alternatives to superparamagnetic metal oxides, having greater superspin magnitudes and lower levels of magnetic disorder. However, synthesis of such nanometals has been hindered by their chemical instability. Here we present a method for preparing air-stable superparamagnetic iron nanoparticles trapped between thermally reduced graphene oxide nanosheets and exhibiting ring-like or core-shell morphologies depending on iron concentration. Importantly, these hybrids show superparamagnetism at room temperature and retain it even at 5 K. The corrected saturation magnetization of 185 Am^2^ kg^–1^ is among the highest values reported for iron-based superparamagnets. The synthetic concept is generalized exploiting functional groups of graphene oxide to stabilize and entrap cobalt, nickel and gold nanoparticles, potentially opening doors for targeted delivery, magnetic separation and imaging applications.

## Abstract (web summary)

Zero-valent metallic nanoparticles can exhibit superparamagnetism, due to quantum effects in magnetic nanomaterials, but their syntheses can be hindered by chemical instability. Here, the authors prepare air-stable superparamagnetic nanoparticles trapped between thermally reduced graphene oxide nanosheets.

Studies on the nanoworld have revealed many new fascinating phenomena and materials with novel physicochemical properties arising from quantum and surface effects^1^. Particularly notable are finite-size effects—quantum phenomena caused by confinement of electron motion in a restricted volume, which gives the system a non-zero lowest energy level and leads to quantization of the available electronic energy levels. Superparamagnetism is a nanoscale phenomenon that originates from finite-size effects in magnetic nanosystems containing transition metals, such as iron, cobalt or nickel^2^,^3^,^4^. The generally accepted model of superparamagnetism assumes *a priori* that a single-domain state is established once the particle size falls below a characteristic threshold value beneath which magnetic domain formation does not reduce the system's overall magnetic energy any longer. Under such conditions, a magnetic nanoparticle can be described in terms of a giant magnetic moment—a superspin—that is equal to a vector sum of all of its atomic and/or ion magnetic moments. As temperature increases, thermal fluctuations become energetically competitive with the particle's magnetic anisotropy. Above a certain threshold temperature, which is determined by the particle's size, thermal fluctuations become dominant and cause the superspin to fluctuate spontaneously between anisotropy-favored orientations. This is known as a superparamagnetic (SP) relaxation, a thermally-driven process that is characterized by the relaxation time between superspin reversals^2^,^3^,^4^. Once the SP regime is established, the superspin can be easily controlled by applying an external magnetic field, causing the system to prioritize anisotropy-preferred orientations that are aligned with the applied field. In real systems, this theoretical picture of superparamagnetism is frequently complicated by factors such as interparticle interactions and surface disorders^5^,^6^.

Together with giant magnetoresistance, superparamagnetism is regarded as one of the eminent nanomagnetic phenomena, and it is considered to have diverse potential applications in practical fields including physics, chemistry, biomedicine and environmental sciences. For example, it was proposed that SP MnAs nanoparticles could be used to create so-called spin batteries in which magnetic energy is converted into electrical energy *via* magnetic quantum tunnelling^7^. In addition, it was demonstrated that micrometer-sized reinforcing particles coated with SP nanoparticles could be used to produce synthetic composites in which the three-dimensional distribution and orientation of reinforcing particles can be tuned by application of small magnetic fields^8^. Superparamagnetism has also been exploited in the construction of self-assembled photonic crystals with stop bands that can be tuned using external magnetic fields, leading to potential applications in colour displays, rewritable signage and sensors^9^,^10^. SP Mn clusters have been used as model systems for studying the quantum-mechanical tunnelling of magnetization in the nanoworld^11^. Most importantly, introduction of SP nanoparticles (especially those based on iron oxides) in various biomedical fields has been proposed to improve efficiency of diagnostic and therapeutic methods minimizing the side effects due to controlled/well-conditioned presence in a living organism and targeted treatment. They have been found effective as contrast agents in magnetic resonance imaging, magnetic carriers for targeted drug delivery and heating elements for the induction of magnetically-assisted hyperthermia^12^,^13^,^14^,^15^,^16^,^17^; some of iron-oxide-based nanosystems were already clinically approved and are used in clinics in magnetic resonance imaging (MRI) and treatment (for example, Lumirem, GastromMARK, Sienna+, Feraheme)^18^.

Iron oxide (Fe_3_O_4_ and γ-Fe_2_O_3_) nanoparticles are the most widely investigated SP nanomaterials due to their low cost, ready availability, numerous optimized synthetic routes and promising biochemical properties (that is, non-toxicity, biodegradability and biocompatibility)^12^,^13^,^14^. They become SP at diameters of <∼15 nm. However, as their size falls below this threshold, the magnitude of their superspin declines markedly due to finite-size effects and formation of magnetically disordered surface layers, limiting their efficiency in practical applications and hampering the development of new ones^5^. Moreover, the net magnetization achievable in these SP materials is determined by the presence of specific magnetically active elements, their distribution within the crystal lattice and strength of associated magnetic exchange interactions, all of which are properties that nanoparticles inherit from their bulk counterparts used in their preparation.

Theory indicates that these drawbacks could potentially be eliminated by replacing metal oxide and alloy nanoobjects with nanoparticles of 3d-block metals such as zero-valent iron, which possess much higher magnetizations that are fully inherited from their bulk forms^19^. Non-interacting magnetic nanometal particles with diameters of <∼5 nm have been predicted to exhibit superparamagnetism^20^, but they are very difficult to synthesize because such small nanometals are unstable under ambient conditions and are rapidly oxidized into respective oxide phases. The only previously reported synthesis of such systems is the preparation of Co/CoO core-shell systems that exhibit SP behaviour at elevated temperatures^21^.

We hypothesize that such metal nanoparticles could be efficiently stabilized if they were trapped in the structure of a suitable host matrix. Moreover, if the matrix were biocompatible, the resulting nanocomposite systems might be viable alternatives to oxide-based nanoparticle assemblies in a range of applications, exhibiting much stronger responses to external magnetic fields and enhanced relaxation. Graphene oxide (GO) was identified as an ideal candidate matrix due to its biocompatibility and ability to host various organic and inorganic species and molecules^22^,^23^,^24^,^25^. Importantly, *in vitro* experiments and *in vivo* cytotoxicity studies showed that GO generally exhibits low cytotoxicity (that is, non-toxic at clinically, diagnostically relevant concentrations up to 500 mg l^–1^) and relatively high cellular uptake, making GO-based materials suitable candidates in various biomedical applications involving cell labelling, intracellular imaging and drug delivery^25^,^26^,^27^,^28^,^29^. Moreover, hybrid materials formed by combining graphene and its derivatives with magnetic nanoparticles could have uses in other fields including energy storage, biosensing, theranostics and environmental remediation^30^. Here, we report (i) the use of GO as a chemical trap enabling metal nanoparticle stabilization (by interactions with oxygen-containing functional groups in the thermally reduced GO structure), (ii) the synthesis of an air- and solution-stable SP nanometals, (iii) potential of free external surface of thermally reduced GO network for secondary functionalization with large surface area and (iv) the experimental (proof-of-concept) demonstration that the iron/GO hybrid system could be viewed as an interesting candidate in MRI applications once its *in vivo* bio-related features are assessed in detail.

## Results

### Physicochemical characterization of developed iron/GO hybrid system

Our synthetic approach is based on impregnation of GO with a suitable metal salt (in the first case, iron nitrate) followed by thermal reduction under a hydrogen atmosphere. This allows the metal content of the resulting hybrid to be specified simply by varying the quantity of metal salt used in the synthesis (for details, see ‘Methods' section). Three composites containing 5, 10 and 20 wt.% of iron embedded in a thermally reduced graphene oxide (TRGO) matrix were prepared and designated Fe(5)/TRGO, Fe(10)/TRGO and Fe(20)/TRGO, respectively. Basic information on the structure, size and morphological arrangements of nanocomposites was obtained by transmission electron microscopy (TEM) and high-resolution transmission electron microscopy (HRTEM) experiments including chemical mapping employing a combined scanning transmission electron microscopy/energy-dispersive X-ray spectroscopy (STEM/EDS) and selected area electron diffraction (SAED) analysis (Fig. 1). Furthermore, magnetization measurements were conducted to characterize the composites' magnetic properties (Supplementary Fig. 1). The microscopic images in Fig. 1 indicate the presence of ultrasmall particles in all the studied hybrids, demonstrating the unique stabilizing properties of the TRGO matrix, however, with clear differences in sizes and structures of iron nanoparticles in each composite that reflect the concentrations of iron nitrate used in their preparation. If the iron concentration is relatively low (5 wt.%), a core-shell architecture is promoted with a core of zero-valent iron and a stabilizing iron(III) oxide shell (Fig. 1a,b). Importantly, the Fe(5)/TRGO hybrid contains ultrasmall SP nanoparticles with diameters below 5 nm, which is consistent with the blocking temperature, *T*_B_, of ∼26 K determined from magnetization measurements (Supplementary Fig. 1a). Presumably, the low iron concentration present during formation of the Fe(5)/TRGO hybrid guarantees that the amount of oxygen liberated from the TRGO matrix is sufficient to enable complete surface oxidation of iron nanoparticles as they form, yielding the observed compact iron(III) oxide shell. The presence of oxidic layer is demonstrated by temperature dependence of the hybrid's magnetization, in particular, the second *T*_B_ at ∼55 K. If the concentration of iron is increased to 10 wt.%, formation of peculiar ring-like assemblies composed of ultrasmall iron nanoparticles (<5 nm) is observed (Fig. 1c,d). No oxidic shell is observed in this case; the rather homogeneous distribution of oxygen seen in the chemical map for the Fe(10)/TRGO hybrid (Fig. 1e,f) corresponds to oxygen-bearing functional groups in the structure of the TRGO matrix. This specific stabilization of SP iron in Fe(10)/TRGO is probably favored because the greater amount of iron relative to the available oxygen prevents formation of a compact iron(III) oxide layer. Following the X-ray photoelectron spectroscopy (XPS) and Raman spectroscopy data analyses (see below), we believe that these nanorings are stabilized by binding interactions between surface Fe(III) species and oxygen-containing functionalities in the TRGO matrix. Magnetization measurements on the Fe(10)/TRGO hybrid indicated that it shows only one *T*_B_ of ∼26 K (Supplementary Fig. 1b), which is consistent with the presence of SP iron nanoparticles with no iron oxide phase. Finally, the use of an even greater concentration of iron during preparation of the Fe(20)/TRGO system yielded larger iron particles (30–50 nm), which again formed ring-like assemblies inside the TRGO matrix (Fig. 1g,h). It appears that at such high iron concentration, the relative concentration of oxygen is too low for oxidic shell formation. The unusual ring-like architecture is probably preserved because iron nanoparticles grow inside cavities that are formed within the TRGO sheets during the thermal process (Supplementary Fig. 2). Unlike the samples prepared with iron loadings of 5 and 10 wt.%, the magnetization data for the Fe(20)/TRGO hybrid do not reveal any evidence of SP behaviour, presumably because of its comparatively large crystals (Supplementary Fig. 1c). In light of its high content of particles below the SP limit and lack of an oxidic shell as well as the unique morphology of its iron nanoparticles, the Fe(10)/TRGO hybrid was selected for further study.

Before performing more detailed analyses of the Fe(10)/TRGO hybrid, samples were subjected to a clean-up procedure involving prolonged sonication followed by filtration. The ‘purification' protocol removed non-embedded and clustered iron nanoparticles from the surface of the hybrid, enabling the isolation of a more pure material comprising only the Fe(10)/TRGO hybrid with embedded SP iron nanoparticles (for details, see ‘Methods' section), preserving their ring-like assemblies. The rings have diameters of 20–100 nm; HRTEM imaging (Fig. 1c,d) revealed that they are made up of ultrasmall nanoparticles with an average diameter of ∼3.5 nm whose size distribution is described by a Gaussian function (see the inset of Fig. 1d). The particles were confirmed to be iron nanoparticles by SAED analysis (see the inset of Fig. 1c, which shows spots clearly assignable to the (110), (200) and (211) planes of α-Fe) and by their measured interplane distance of 2.86 Å, which corresponds to the (100), (010) or (001) crystal planes of the body-centered-cubic (bcc) structure of α-Fe (see the inset of Fig. 1d). The chemical composition of the Fe(10)/TRGO hybrid and chemical bonds present in the system were investigated by XPS and Raman spectroscopy. The survey XPS spectrum recorded for the Fe(10)/TRGO hybrid together with atomic adsorption spectroscopy (AAS) analysis confirm the presence of iron species amounting to ∼10 wt.% in the sample. The high-resolution C1s XPS pattern of the Fe(10)/TRGO hybrid (Supplementary Fig. 3a) shows a relatively low level of oxidation, as expected for TRGO^31^, with dominating C–C (*sp*^2^) (at 284.74 eV) and C–C (*sp*^3^) (at 285.57 eV) peaks, which together account for almost 80% of the spectral area. The dominant oxygen-bearing groups feature C–O and C=O bonds; O–C=O groups contribute rather marginally. The C1s XPS spectrum of the Fe(10)/TRGO hybrid contains no evidence of Fe–C bonding. In contrast, not only the high-resolution O1s XPS pattern of the Fe(10)/TRGO hybrid (Supplementary Fig. 3b) exhibits evidence of the expected C–O and C=O bonds but also of Fe–O bonds with a binding energy of 530.5 eV^32^. Because the intensity of this peak is very low, it can be attributed to a partial stabilization and oxidation of the surface iron atoms *via* interactions with oxygen atoms belonging to functional groups of the TRGO matrix. The Raman spectrum of the Fe(10)/TRGO hybrid is shown in Supplementary Fig. 4. The peaks at 1,345, 1,580, 2,663 and 2,927 cm^–1^ are typical of TRGO, and were assigned to the D, G, 2D and D+G bands, respectively^33^. Most importantly, the intensity of the 2D peak is much lower than that of the G peak, indicating that the TRGO nanosheets of the hybrid material are few-layered. The space restrictions imposed by the few-layered architecture combined with the stabilizing effects of the TRGO's oxygen functionalities are presumably important in enabling the entrapment of the iron nanoparticles and the preservation of their chemical and morphological properties even at room temperature. The presence and stabilization of iron nanoparticles are evidenced by the peaks at 490 and 592 cm^–1^, which can be assigned to Fe–O bonds^34^ in accordance with XPS data.

^57^Fe Mössbauer spectroscopy was then used to investigate the structural and magnetic features of the Fe(10)/TRGO nanocomposite in more details. The room-temperature ^57^Fe Mössbauer spectrum of the Fe(10)/TRGO hybrid is dominated by a singlet with a zero isomer shift (Fig. 2a; Supplementary Table 1), indicating that the ultrafine α-Fe nanoparticles in the hybrid material are in the SP state at room temperature and within the measuring time window of the Mössbauer technique (∼10^–8^ s). At 50 K, a sextet emerges in addition to the singlet component (Fig. 2b); the hyperfine Mössbauer parameters for this sextet also correspond to α-Fe (Supplementary Table 1). The appearance of sextet component is attributed to the magnetic blocking of some α-Fe nanoparticles. As the temperature is lowered further, the spectral area of the sextet increases at the expense of that for the singlet (Fig. 2c; Supplementary Table 1), which is typical for a system with magnetic nanoparticles of varied sizes undergoing a transition from the SP regime to a magnetically blocked regime. However, the singlet persists even at 5 K, demonstrating that the superspins of the smallest iron nanoparticles continue to exhibit SP fluctuations even at this low temperature, a feature that has never previously been observed for any metal/metal oxide/metal alloy nanoparticles. Remarkably, Mössbauer hyperfine parameters derived from the sextet component at 5 K are practically identical to those frequently reported for bulk α-Fe (isomer shift, *δ*, of 0.12 mm s^–1^, quadrupole splitting, Δ*E*_Q_, of 0.00 mm s^–1^ and hyperfine magnetic field, *B*_hf_, of 33.1 T). In particular, zero quadrupole shift and negligible decrease in *B*_hf_ indicate a high degree of symmetry in the local environment of the iron nuclei and the presence of a fully developed magnetic structure, respectively. This implies that finite-size and surface effects have less influence on the physical properties of the nanoparticles in the hybrid material than they do in comparably sized iron oxide nanoparticles^1^. Ultrafine iron nanoparticles with sizes of ∼2 nm whose ^57^Fe Mössbauer spectra feature singlets at low temperatures (50 K) were reported by Bodker *et al.*^35^, Margeat *et al.*^36^ and Lacroix *et al.*^37^. However, none of these systems were shown to be air-stable and they would probably be rapidly converted into iron oxide phases on exposure to air. Importantly, the relative spectral area of the Fe(III) doublet component is ∼20% in all of the ^57^Fe Mössbauer spectra of the Fe(10)/TRGO hybrid (Fig. 2), indicating that the SP/paramagnetic behaviour of the Fe(III) species in the hybrid remains constant over the entire studied temperature interval, which has never previously been observed for any iron(III) oxide phase of crystalline or amorphous origin^38^,^39^. This is further evidence that the octahedrally coordinated Fe(III) ions present in this system form bonding interactions with oxygen functionalities in the TRGO matrix that chemically stabilize iron nanoparticles.

The remarkable magnetic properties of the Fe(10)/TRGO nanocomposite were further studied by performing magnetization measurements. At 5 K, the hysteresis loop of the Fe(10)/TRGO hybrid shows a non-zero coercivity and remanence (Fig. 3a), indicating that a majority of the iron nanoparticles are in a magnetically blocked state. The uniform arrangement of all the atomic magnetic moments inside the nanoparticles is demonstrated by the saturation of the hybrid material's magnetization by applied fields as weak as ∼1 T (Fig. 3a). The saturation tendency of iron nanoparticles under weak applied magnetic fields is surprising in contrast to the behaviour of metal oxide (iron oxide) nanoparticles with similar average particle sizes, which generally do not exhibit complete magnetic saturation even under applied fields of up to 5 T (that is, the applied field is not strong enough to overcome the effects of the iron oxide nanoparticles' local and surface magnetic anisotropies, which imprint specific and more energetically favourable orientations on the magnetic moments of the atoms around the defects and in the surface layers of the nanoparticles). This implies that the surface magnetic anisotropy of the iron nanoparticles in the Fe(10)/TRGO hybrid material is much smaller than that in iron oxide nanoparticles of similar size. As the temperature is raised, superspins of iron nanoparticles gradually become unblocked and enter the SP regime. At 300 K, no hysteresis is observed (Fig. 3a), meaning that all of the magnetic nanoparticles in the hybrid material are in the SP state within the time scale of the magnetization measurements (∼10 s). This conclusion is further supported by the zero-field-cooled (ZFC)/field-cooled (FC) magnetization curves; the ZFC magnetization curve shows a maximum at around 26 K, which corresponds to average *T*_B_ for iron nanoparticles of the most abundant size (Fig. 3b). The two curves diverge at around 40 K (Fig. 3b), which corresponds to the so-called irreversibility temperature, *T*_irr_, that is, the temperature at which the largest iron nanoparticles in the system enter the low-temperature magnetically blocked regime. The difference between *T*_B_ and *T*_irr_ can be regarded as a quantitative measure of the particle size distribution; the small difference between these values indirectly suggests a narrow particle size distribution in agreement with TEM data. Thus, the TRGO matrix is a very efficient trap for stabilizing ultrasmall nanoparticles and preventing their growth. There is no observable magnetic blocking of the Fe(III) environment, which interacts directly with the TRGO matrix. This excludes the possibility that the hybrid material contains iron oxide phases because such phases are always magnetically ordered at 5 K, even in the case of ultrasmall amorphous nanoparticles/shells. If the magnetization values are recalculated to reflect the contribution of iron to the total mass of the hybrid material and the magnetic response of TRGO is subtracted, the nanoparticles' saturation magnetization, *M*_S_, is almost 185 Am^2 ^kg^–1^ at 300 K, one of the highest values observed in the SP state for any metal-oxide-based or alloy-based system. Remarkably, for such small iron nanoparticles, the *M*_S_ value is only ∼15% lower than that of bulk α-Fe (∼215 Am^2^ kg^–1^). As a result of a high magnetization at room temperature, the Fe(10)/TRGO hybrid responds strongly even to simple hand-held magnets (Supplementary Fig. 5), which could be extremely useful for magnetic targeting and separation in biomedical and environmental applications.

The results imply that in the Fe(10)/TRGO composite, finite-size and surface effects do not significantly affect the magnetic response of the entrapped iron nanoparticles. Conversely, metal oxide nanoparticles^5^ exhibit markedly reduced *M*_S_ values and a strong tendency towards non-saturation of magnetization in high applied fields as their size is reduced. As predicted by theoretical studies^40^, differences in the influence of finite-size and surface effects can be understood by considering the distinct mechanisms that give rise to magnetic ordering in metals and their oxides, and the way in which electrons occupy available electronic energy levels in the clusters^19^. For metal oxide nanoparticles, atomic magnetic moments are ordered *via* superexchange interactions in which oxygen orbitals serve as mediators between magnetically active atoms. As the particle size of metal oxides is reduced, the strength of these magnetic bonds declines because the corresponding chemical bonds are weakened and there is more pronounced symmetry breaking in the nanoparticle's surface layers. Both of these effects are manifested in lower magnetization values^5^. In contrast, the magnetic ordering of metal nanoparticles is governed by (i) direct exchange interactions if there is direct overlap between localized electronic orbitals on adjacent magnetically active sites and (ii) Ruderman–Kittel–Kasuya–Yosida (RKKY) interactions in which conduction electrons serve as mediators of magnetic interactions between atomic magnetic moments. Iron nanoparticles entrapped in the TRGO matrix are not subject to marked weakening of RKKY interactions with decreasing particle size, retaining thus high *M*_S_ values. Moreover, the superspin of metal nanoparticles may even increase as they get smaller because electrons become increasingly likely to occupy configurations that favour unpaired atomic spins^41^.

### Proof-of-concept demonstration of iron/GO hybrid system in MRI

To demonstrate the bio-applicability of the Fe(10)/TRGO, we performed additional analyses and post-treatment experiments. Importantly, the chemical nature (and hence, magnetic features) of entrapped iron nanoparticles was stable to prolonged storage (30 days) in air or a physiological solution as demonstrated by the ^57^Fe Mössbauer spectra (Supplementary Fig. 6; Supplementary Table 2). For potential bio-applications, the Fe(10)/TRGO nanocomposite was modified with polyethylene glycol (PEG), which is commonly used for surface functionalization of carbon-based nanomaterials to increase their hydrophilicity and biocompatibility^25^. As can be clearly seen in Supplementary Fig. 7, PEGylation drastically increased the colloidal stability of the Fe(10)/TRGO hybrid in both physiological and acidic solutions.

To assess the biocompatibility of the Fe(10)/TRGO and Fe(10)/TRGO/PEG systems, standard viability experiments based on the MTT assay were performed using NIH/3T3 mouse fibroblasts (Fig. 4a). Neither dispersion exhibited any discernible toxicity towards tested cells at concentrations up to 250 μg ml^–1^, implying that both hybrid systems can be viewed as non-toxic in terms of *in vitro* and *in vivo* clinically, diagnostically relevant concentrations. In addition, we performed in parallel microscopic analysis of the cells labelled with the same concentrations of Fe(10)/TRGO/PEG particles as used in the MTT assay. We did not observe any significant changes in the cell morphology, proliferation or deadheration of cells during the 24 h compared with control cells (Supplementary Fig. 8).

These results show that the PEGylated Fe(10)/TRGO hybrid is chemically and colloidally stable, hydrophilic, biocompatible and does not cause any *in vitro* toxic effects at relatively high concentrations. All of these factors support its potential utility as an MRI contrast agent for improving the quality of *T*_2_-weighted images. Because *T*_2_ spin–spin relaxation times depend on the magnitude of the magnetic moment among other things, the high saturation magnetization of entrapped iron nanoparticles in the Fe(10)/TRGO/PEG hybrid should encourage negative contrast properties. Indeed, when employing a 9.4 T MRI scanner, the hybrid exhibited a much higher *r*_2_ relaxivity (153 mM^–1^ s^–1^) than was achieved with FeraSpin XXL, the commonly used commercial SP iron oxide (SPIO)-based *T*_2_ contrast agent (64.3 mM^–1^ s^–1^, Supplementary Fig. 9a). Importantly, the ratio of *r*_2_/*r*_1_ relaxivities for the Fe(10)/TRGO/PEG system was calculated to be 728. Such a high *r*_2_/*r*_1_ ratio greatly enhances negative contrast properties in *T*_2_-weighted imaging compared with those exhibited by the commercial FeraSpin XXL agent (see the phantom experiment results in Supplementary Fig. 9c). To compare its contrast features to those of other previously clinically approved MRI contrast agents, the *r*_1_ and *r*_2_ relaxivities for Fe(10)/TRGO were also measured under a field of 4.7 T and compared with reference values from the literature (Supplementary Fig. 9b; Supplementary Table 3)^42^. This analysis yielded *r*_2_ and *r*_2_/*r*_1_ values of 163 mM^–1^ s^–1^ and 398 mM^–1^ s^–1^, respectively, which are comparable to those of non-SPIO currently used MRI contrast agents^42^ and higher than those reported for any SPIO-based contrast agent previously clinically approved in MRI diagnostics (for example, Lumirem, GastromMARK, Sienna+, Feraheme, Resovist, Feridex and so on)^18^,^37^. Moreover, the relaxivity characteristics observed for the Fe(10)/TRGO hybrid are broadly comparable to the most advanced metal-oxide- or metal-alloy-based systems that have been reported in the literature and are in the pre-clinical stage (before potential clinical approval)^43^,^44^,^45^.

On the basis of these promising *in vitro* results, we performed a preliminary (proof-of-concept) *in vivo* MRI experiment with the Fe(10)/TRGO/PEG composite. Before *in vivo* application, we checked the hydrodynamic size of the Fe(10)/TRGO/PEG system by optical microscopy (Supplementary Fig. 10); it is clearly seen that in the sample after PEGylation, sonication and size fractionation by weak centrifugation, particles of sizes of <1 μm appear, stable in phosphate-buffered saline (PBS), which can be used for safety intravenous applications (according to the veterinary rules). Then, after intravenous administration into the tail vein of a healthy mouse, we monitored the hybrid's bio-distribution and contrast effects using a 9.4 T MR scanner (for details, see ‘Methods' section). A significant decrease in the signal intensity was observed within a few minutes of hybrid administration, primarily in the liver and kidneys (Fig. 4b,c). This is consistent with the behaviour observed with most frequently used iron-oxide-based intravenous contrast agents for MRI. Here, we stress that these data provide just preliminary information on potential applicability of the Fe/TRGO systems in MRI and definitely, further detailed *in vitro*/*in vivo* studies assessing a complex bio-related features of the hybrid such *in vitro*/*in vivo* stability, toxicity, bio-distribution and bio-half time are highly required in future.

### Generalization of the concept of preparing air-stable nanometals with GO

Finally, the potential for extending the concept of thermally induced entrapment in few-layered TRGO sheets to other metals was tested by preparing Co(10)/TRGO and Ni(5)/TRGO nanocomposites with 10 and 5 wt.% of cobalt and nickel inside TRGO, respectively, as checked by the AAS technique. Figure 5a,b show selected TEM/HRTEM images of the resulting Co(10)/TRGO hybrids, which feature ring-like superstructures composed of ultrasmall cobalt nanoparticles that closely resemble those seen in the Fe(10)/TRGO system. The material's measured interplane distance of 2.50 Å corresponds well to (100) or (010) crystal planes of cobalt. Nanoparticles have similar dimensions (below 6 nm) to those of the Fe(10)/TRGO hybrid and exhibit SP behaviour at room temperature (with *T*_B_ at ∼22 K, Supplementary Fig. 11). The predominant nanostructures observed in the Ni(5)/TRGO hybrid were core-shell structures with nickel nanoparticle cores and stabilizing NiO shells (Fig. 5c–e), like those seen in the Fe(5)/TRGO nanocomposite. Importantly, nickel nanoparticles were ultrasmall (<6 nm) and showed the expected room-temperature SP characteristics with *T*_B_ of ∼15 K (Supplementary Fig. 12). The slightly lower *T*_B_ for entrapped SP nickel compared with SP iron nanoparticles of comparable size is consistent with the lower magnetic hardness of nickel.

These results clearly confirm the universality of our approach for preparing metal nanoparticles by chemical impregnation of GO with a suitable metal salt followed by thermal reduction to achieve effective entrapment and stabilization of SP (iron, cobalt, nickel) nanometals inside the TRGO matrix (Fig. 6). Three factors appear to be crucial for their stabilization and controlling the morphological arrangement of resulting nanoparticles: (i) spatial restrictions on nanoparticle growth imposed by the few-layered TRGO matrix; (ii) oxygen functionalities of the TRGO matrix, which act as chemical traps that stabilize the nanoparticles by forming chemical bonds with surface metal atoms; (iii) initial concentration of metal in the system, which is important because it determines the metal-to-oxygen ratio, and thereby controls the size and morphological arrangement of the formed nanoparticles, dictating formation of core-shell or nanoring structures. In addition, free external surface of TRGO network with large surface area offers a secondary functionalization with biomolecules and/or drugs.

Importantly, the presented method for nanometal entrapment appears to be very general: it can also be used to prepare ultrasmall noble metal nanoparticles (below 5 nm) if a suitable precursor salt is used, as demonstrated by the synthesis of an Au(10)/TRGO nanocomposite (Fig. 5f–h) with 10 wt.% of gold trapped inside the TRGO matrix as checked by the AAS technique. In such cases, the TRGO matrix presumably only imposes spatial restriction with no chemical stabilization of the noble metal.

## Discussion

We developed a universal method for the synthesis of ultrasmall metal (iron, cobalt, nickel) nanoparticles that exhibit SP behaviour even at room temperature over a wide range of time scales (from 10^–8^ to 10 s). The metal nanoparticles are grown and entrapped inside a few-layered two-dimensional TRGO matrix, where they are stabilized by interactions with oxygen-containing functional groups in the TRGO structure. By varying the initial concentration of the metal salt used in the synthesis, it is possible to obtain metal nanoparticles with either ring-shaped superstructures or core-shell architectures. If placed in an external magnetic field, the Fe/TRGO material exhibits a strong magnetic response, with the iron nanoparticles' saturation magnetization reaching almost 185 Am^2^ kg^–1^ even under a 1 T field. A PEG-functionalized Fe/TRGO hybrid exhibited enhanced colloidal stability and *in vitro* biocompatibility, and proved to be a promising powerful *T*_2_ negative contrast agent for MRI, with contrast properties comparable to or better than most commercially used MRI agents.

We believe that TRGO trapping is a generally applicable method for the synthesis of nanometals and alloys (for example, FePt nanoparticles) with particle sizes and morphologies that can be controlled by careful selection of metal precursors that are used and their concentrations. This could facilitate development of new nanotechnologies that exploit entrapped SP nanometals for MRI and targeted drug delivery or to create energy materials (spin batteries) and sensors. Moreover, this method provides a space to expand the diverse applications of TRGO by enabling the preparation of TRGO derivatives that have clean surfaces while still enabling magnetic separation and reusability.

## Methods

### Samples preparation

Firstly, GO was synthesized similarly to the Hummers method. Graphite (Sigma-Aldrich, 5g) and sodium nitrate (Sigma-Aldrich, 2.5g) were stirred with sulphuric acid (Sigma-Aldrich, 98%, 115ml). The mixture was then cooled to 0°C. Potassium permanganate (Sigma-Aldrich, 15g) was then added over a period of 2h. During next 4h, the reaction mixture was allowed to reach room temperature before heating to 35°C for 30min. The reaction mixture was then poured into a flask containing deionized water (250ml) and heated to 70°C for 15min. The mixture was then poured into deionized water (1l). The unreacted potassium permanganate and manganese dioxide were removed by the addition of 3% hydrogen peroxide (Sigma-Aldrich). The reaction mixture was then allowed to settle and decant. The obtained GO was then purified by repeated centrifugation and redispersing in deionized water until a negative reaction on sulphate ions was achieved. GO slurry was then dried for 48h in a vacuum oven at 50°C. A sample containing iron nanoparticles trapped in a TRGO matrix was then prepared by the thermal treatment of GO (200 mg), impregnated with Fe(NO_3_)_3_·9H_2_O (Sigma-Aldrich; 159 mg, that is, 10 wt.%) under an atmosphere of hydrogen. The resulting mixture was then dried in a vacuum oven at 50 °C for 48 h, after which the dried nanocomposite was placed inside a quartz glass capsule connected to a magnetic manipulator. The loaded capsule was placed inside a horizontal quartz glass reactor that was repeatedly evacuated and flushed with nitrogen. The nitrogen atmosphere in the reactor was then replaced with hydrogen and the sample was transferred to the reactor's hot zone, where it was heated at 1,000 °C for 10 min under an atmosphere of pure H_2_ (1 bar pressure). Finally, a hydrogen flow of 1,000 ml min^–1^ was used to remove the gaseous by-products of the reaction process. After the reaction procedure, the composite, denoted as Fe(10)/TRGO, was removed from the hot zone and the entire apparatus was flushed with nitrogen before being opened. The same synthetic procedure was used to prepare the hybrids with different concentration of iron in the TRGO matrix as well as nanocomposites consisting of TRGO matrix with cobalt, nickel and gold nanoparticles entrapped inside. The samples are denoted as Fe(5)/TRGO, Fe(20)/TRGO, Co(10)/TRGO, Ni(10)/TRGO and Au(10)/TRGO. For the synthesis of hybrids with different iron concentration, the identical starting weight of GO was kept as in the case of the Fe(10)/TRGO sample, while the weight of Fe(NO_3_)_3_·9H_2_O precursor changed to 80 and 318 mg to obtain Fe(5)/TRGO and Fe(20)/TRGO hybrid, respectively. For the synthesis of the hybrids with 10 wt.% of Co, 5 wt.% of nickel and 10 wt.% of Au in the TRGO matrix, Co(NO_3_)_2_·6H_2_O (Sigma-Aldrich) precursor (109 mg), Ni(NO_3_)_2_·6H_2_O (Sigma-Aldrich) precursor (55 mg) and AuCl_3_·3H_2_O (Sigma-Aldrich) precursor (37 mg) were used keeping the identical weight amount of GO respectively.

The Fe(10)/TRGO nanocomposite was further purified by post-processing treatment because ^57^Fe Mössbauer spectroscopy indicated that the unpurified reaction product involved three iron-containing fractions (Supplementary Table 1): (i) ultrasmall SP iron nanoparticles embedded in the TRGO matrix that give rise to a singlet component in the room-temperature ^57^Fe Mössbauer spectrum, (ii) larger ferromagnetic/magnetically blocked iron nanoparticles that presumably formed on the air-reachable surfaces of the TRGO nanosheets and give rise to a sextet component and (iii) iron(III) species covering the surfaces of the larger iron nanoparticles, which interact with oxygen atoms from TRGO matrix and give rise to a doublet. To release the weakly bound larger ferromagnetic iron nanoparticles formed on the surface of the TRGO sheets network, the Fe(10)/TRGO hybrid was re-dispersed in distilled water (1 mg ml^–1^) and sonicated in an ultrasound bath for 5 min. The resulting dispersion was filtered through a Millipore syringe filter (200 nm) to remove the liberated larger nanoparticles while trapping the Fe(10)/TRGO hybrid, which was then re-dispersed in water, centrifuged and dried under vacuum.

To increase biocompatibility and hydrophilicity, the surface of the Fe(10)/TRGO hybrid was non-covalently stabilized by PEG 3,000 (O-(2-aminoethyl)polyethylene glycol) from Sigma-Aldrich. Briefly, before PEGylation process, we applied a secondary more intensive (50 kHz) and prolongated (2 h) sonication to release and remove all the Fe/Fe(III) species attached to the surface. Then, 15 mg of Fe(10)/TRGO nanocomposite was mixed with 15 mg of PEG in 15 ml of water and sonicated in ultrasound bath for 4 h. The prepared Fe(10)/TRGO/PEG hybrid was four times centrifuged at 10,000*g* for 30 min and re-dispersed in water and physiological solution for subsequent *in vitro* and *in vivo* study.

### Characterization techniques

The concentration of iron, cobalt, nickel and gold in the respective hybrid material was determined by AAS technique with flame ionization using a ContrAA 300 instrument (Analytik Jena AG, Germany) equipped with a high-resolution Echelle double monochromator having a spectral bandwidth of 2 pm at 200 nm and a continuum radiation source (xenon lamp). The absorption line at 248.3, 240.7, 232 and 242.8 nm was used for iron, cobalt, nickel and gold analysis. TEM/HRTEM was used to conduct particle size measurements and morphological studies of solid samples. All the TEM experiments were performed with a JEOL JEM-2010 TEM equipped with a LaB_6_ cathode operated at an accelerating voltage of 160 kV with a point-to-point resolution of 0.194 nm. A drop of high-purity distilled water was placed onto a holey carbon film supported on a copper-mesh TEM grid (SPI Supplies, USA) and air-dried at room temperature. The dimensions of the nanoparticles were measured using the ITEM programme. HRTEM images were obtained using a HRTEM TITAN 60–300 microscope with an X-FEG type emission gun, operating at 300 kV. This instrument is equipped with a Cs image corrector and a STEM/HAADF detector; its point resolution is 0.06 nm in the TEM mode. Elemental mappings were obtained by STEM/EDS technique with an acquisition time of 20 min. For HRTEM analyses, powder samples were dispersed in ethanol and ultrasonicated for 5 min. One drop of the resulting suspension was then placed on a copper grid covered with a holey carbon film and allowed to dry at room temperature. XPS measurements were carried out with a PHI VersaProbe II (Physical Electronics) spectrometer using an Al K_α_ source (15 kV, 50 W). All spectra were acquired under a partial vacuum (1.4 × 10^–7^ Pa) at room temperature (22 °C). High-resolution C1s and O1s XPS patterns were acquired by setting the pass energy to 23.500 eV and the step size to 0.200 eV. The XPS patterns were analyzed using the MultiPak (Ulvac—PHI) programme. All binding energy values were referenced to the C1s peak at 284.80 eV. Raman spectra were collected using a DXR Raman spectroscope (Thermo Scientific, USA) equipped with a laser operating at a wavelength of 532 nm. The laser power on the sample was set to 2 mW. Each measured Raman spectrum was an average of 32 experimental microscans. The acquisition time was set to 1 s. Transmission ^57^Fe Mössbauer spectra were acquired using a Mössbauer spectrometer operating in a constant acceleration mode and equipped with a 50 mCi ^57^Co(Rh) source. For low-temperature measurements, the samples were placed inside the chamber of a cryomagnetic system (Oxford Instruments, UK). The ^57^Fe Mössbauer spectra were then fitted using the MossWinn programme; before fitting, the signal-to-noise ratio was enhanced using a statistical approach that combines routines incorporated into MossWinn software package and the procedures developed by Prochazka *et al.*^46^. Isomer shift values are referenced to data for α-Fe foil at room temperature. A superconducting quantum interference device (SQUID)-based magnetometer (MPMS XL-7 type, Quantum Design, USA) was employed for magnetization measurements. The hysteresis loops of all the studied samples were measured at temperatures of 5 and 300 K under external magnetic fields ranging from −5 to+5 T. The ZFC and FC magnetization curves were recorded on warming in the temperature range from 5 to 300 K and in an external magnetic field of 0.1 T after cooling in a zero magnetic field and a field of 0.1 T, respectively.

### *In vitro* cytotoxicity study and *in vitro* MRI measurements

The toxicity of the Fe(10)/TRGO and Fe(10)/TRGO/PEG hybrid materials was tested using the MTT assay with the NIH/3T3 mouse fibroblasts purchased from the American-type Culture Collection (ATCC, USA). The fibroblasts were cultivated in DMEM growth medium (low glucose Dulbecco's Modified Eagle medium, Lifetechnologies) at 37 °C under a CO_2_-enriched (5%) atmosphere. The material's effects on cellular viability were assessed by preparing a dilution series in ultrapure water at concentrations of 1–200 μg ml^–1^. Cells in DMEM media were seeded into a 96-well plate and left for 3 h to spread, after which they were treated with Fe(10)/TRGO and Fe(10)/TRGO/PEG suspensions at various concentrations in ultrapure water and incubated for 24 h. A solution of MTT (3-(4,5-dimethylthiazol-2-yl)-2,5-diphenyltetrazolium bromide) in water was then added to each well (20 μl, 5 mg ml^−1^). After incubation for 24 h, the MTT solution was removed and dimethylsulfoxide (100 μl) was added to dissolve the resulting formazan crystals. The absorbance of the solutions formed in this way was measured at 570 nm using an Infinite PRO M200 multiplate reader (Tecan, Austria). The cytotoxicity of tested Fe(10)/TRGO and Fe(10)/TRGO/PEG nanocomposites was determined by comparing the absorbances of the treated samples to those of an untreated control and plotting the resulting ratios as viability percentages given by the expression (*A*_sample_/*A*_control_) × 100. Both suspensions were assayed in triplicate within each run of the experiment, and two duplicate experimental runs were performed.

MRI measurements were performed with a 4.7 T (MR6000 spectrometer by MR Solutions, UK, 4.7 T/200 mm superconducting magnet by Magnex Scientific, UK, 1 kW RF amplifier of 5T1000M type by CPC Amps, USA, GPA 200–350 gradient amplifiers from International Electric Company, Finland) and a 9.4 T (Bruker-BioSpec 94/30 USR, Ettlingen, Germany) NMR system. Six 0.5 ml samples of agar gel mixed with the Fe(10)/TRGO nanocomposite with concentrations of 33, 50, 125, 250, 500 and 750 μM Fe were measured. The samples were measured in the 2-ml Eppendorf microtubes. For a comparison, a commercial contrast agent, FeraSpin XXL (Miltenyi Biotec, Bergisch Gladbach, Germany) was also measured; it was mixed with 1.5% agar gel to yield concentrations of 0, 33, 50, 125 and 250 μM. The 1.5 ml samples were measured in 1.5 ml Eppendorf microtubes. All the measurements were performed at the laboratory temperature.

For the Fe(10)/TRGO hybrid sample in the 9.4 T NMR scanner, images for *T*_1_ and *T*_2_ quantification were acquired using a rapid acquisition with refocused echoes (RARE) pulse sequence (TR=27–12,000 ms; TE=10–150 ms, RARE factor=2, 256 × 256 matrix) and for *T*_2_* quantification, multiple gradient echo (MGE) pulse sequence (TR=12,000 ms, TE=4–124 ms, flip angle=30°, 256 × 256 matrix) was used. For FeraSpin XXL and for *T*_2_ quantification, the RARE pulse sequence (TR=15,000 ms, TE=11–176 ms, 128 × 128 matrix) was used. Slice thickness (SL) for all acquisitions was 1 mm, FOV=6 × 4 cm and single slice was used. The values of *T*_1_, *T*_2_ and *T*_2_* were calculated for each sample in manually drawn regions of interest (ROIs) using the image sequence analysis tool (ParaVision v.5.1, Bruker BioSpin, Ettlingen, Germany).

Using the 4.7 T NMR system, four samples of the Fe(10)/TRGO hybrid were measured (concentrations of 31, 63, 125 and 250 μM Fe). A spin echo (SE) pulse sequence was applied in image acquisition for *T*_1_ quantification (TR=22–15,000 ms, TE=13 ms) and *T*_2_ quantification (TR=12,000 ms, TE=13–150 ms). A gradient echo (GE) pulse sequence was applied in image acquisition for *T*_2_* quantification (TR=12,000 ms, TE=9–50 ms, FA=50°). For all the acquisitions, SL=1 mm, FOV=4 × 4 cm and matrix=64 × 64. The signal intensity within the hand-drawn ROIs were extracted using the MAREVISI software (National Research Council Canada, Ottawa) and the relaxation times were then estimated using own software implemented in MATLAB (MathWorks, Natick, USA).

Finally, the *r*_1_, *r*_2_ and *r*_2_* relaxivities were calculated as proportionality constants of the linear relation between the reciprocal relaxation time and the contrast-agent concentration.

### *In vivo* MRI study

The *in vivo* MRI experiments with a healthy mouse (35 g, male, ICR) were performed at 9.4 T employing a 9.4 T NMR system (Bruker-BioSpec 94/30 USR, Ettlingen, Germany). The animal procedure was in accordance with the European Community's Council Directive (2013/148/EEC) and approved by the Ethics Committee of The Czech Academy of Sciences in compliance with the Czech Animal Protection Act No. 246/1992. The Fe(10)/TRGO/PEG hybrid was administered intravenously with a dose of 10 mg of Fe per kg of mouse body weight. To monitor the bio-distribution and the effect of the contrast agent on MRI intensity in the *T*_2_-weighted images, MSME sequence (TR=2,500 ms, TE=36 ms, SL=1.42 mm, acquisition time=4 min) and MGE sequence (TR=22.9 ms, TE=5 ms, SL=1.42 mm, FA=14°, 2 segments, respiration gating) were used.

### Data availability

The data that support the findings of this study are available from the corresponding author upon request.

## Additional information

**How to cite this article:** Tuček, J. *et al.* Air-stable superparamagnetic metal nanoparticles entrapped in graphene oxide matrix. *Nat. Commun.* 7:12879 doi: 10.1038/ncomms12879 (2016).

## Supplementary Material

Supplementary Information Supplementary Figures 1-12 and Supplementary Tables 1-3

Peer review file

## Figures and Tables

**Figure 1:** Electron microscopy and chemical mapping of the nanocomposites. (**a**) Representative TEM image (scale bar, 50 nm) of the Fe(5)/TRGO hybrid system with the inset showing a magnified HRTEM image (scale bar, 5 nm) of a single iron nanoparticle with a core-shell structure. (**b**) STEM/EDS chemical mapping (Fe and O; scale bar, 4 nm) of a single iron nanoparticle in the Fe(5)/TRGO nanocomposite. (**c**) Representative TEM image (scale bar, 50 nm) of the Fe(10)/TRGO hybrid system with the inset showing the SAED pattern. (**d**) Representative HRTEM image (scale bar, 20 nm) of the Fe(10)/TRGO hybrid system demonstrating the ring-link assembly of iron nanoparticles inside the TRGO matrix with insets showing a single iron nanoparticle with marked atomic layers separated by 2.86Å (scale bar, 5 nm) and the particle size distribution. (**e**) High-angle annular dark-field (HAADF) images (scale bar, 20 nm) of the Fe(10)/TRGO nanocomposite. (**f**) STEM/EDS chemical mapping (Fe and O; scale bar, 4 nm) of a single iron nanoparticle in the Fe(10)/TRGO hybrid system. (**g**) Representative TEM image (scale bar, 200 nm) of the Fe(20)/TRGO nanocomposite with the inset (scale bar, 20 nm) showing the ring-like arrangement of iron nanoparticles inside the TRGO matrix. (**h**) Representative HRTEM image (scale bar, 20 nm) of the Fe(20)/TRGO hybrid system with the inset showing STEM/EDS chemical mapping (Fe; scale bar, 10 nm) of iron nanoparticles in their ring-like assembly.

**Figure 2:** ^57^Fe Mössbauer spectra of the Fe(10)/TRGO nanocomposite. ^57^Fe Mössbauer spectra acquired at temperatures of (**a**) 300 K, (**b**) 50 K and (**c**) 5 K.

**Figure 3:** Magnetization measurements of the Fe(10)/TRGO nanocomposite. (**a**) Hysteresis loops of the Fe(10)/TRGO nanocomposite, recorded at a temperature of 5 and 300 K, with the insets showing the behaviour of hysteresis loops in weak applied fields and hysteresis loops recalculated with respect to the proportion (by mass) of iron nanoparticles in the TRGO network. (**b**) ZFC/FC magnetization curves of the Fe(10)/TRGO nanocomposite with insets showing the profile of the ZFC/FC magnetization curves at low temperatures and a schematic illustration of the blocked and SP states of self-assembled iron nanoparticles trapped inside the TRGO network.

**Figure 4:** Biocompatibility tests and *in vivo* MRI measurements. (**a**) Viability of cells exposed to the Fe(10)/TRGO and the Fe(10)/TRGO/PEG nanocomposite determined by the MTT assay (data presented are the mean±s.d. of triplicate assays). (**b**) Schematic image of the mouse's abdominal region with marked organs. (**c**) *In vivo* MRI images of a healthy mouse in the coronal plane, collected before and after intravenous injection of the Fe(10)/TRGO/PEG nanocomposite, showing clearly the reduction in the signal intensity for the kidneys and liver in the *T*_2_-weighted MRI images.

**Figure 5:** Characterization of the nanocomposites containing other metals. (**a**) Representative TEM image (scale bar, 50 nm) of the Co(10)/TRGO hybrid system with the inset (scale bar, 5 nm) showing a single cobalt nanoparticle with marked atomic layers separated by 2.50Å. (**b**) Representative HRTEM image (scale bar, 10 nm) of the Co(10)/TRGO hybrid system demonstrating the ring-like arrangement of cobalt nanoparticles inside the TRGO matrix. (**c**) Representative HRTEM image (scale bar, 20 nm) of the Ni(5)/TRGO hybrid system. (**d**) HAADF image (scale bar, 6 nm) of a single nickel nanoparticle in the Ni(5)/TRGO nanocomposite. (**e**) STEM/EDS chemical mapping (Ni and O; scale bar, 6 nm) of the Ni(5)/TRGO hybrid system demonstrating the core-shell architecture of the trapped nickel nanoparticle inside the TRGO network. (**f**) Representative HRTEM image (scale bar, 20 nm) of the Au(10)/TRGO nanocomposite. (**g**) HAADF image (scale bar, 4 nm) of a single gold nanoparticle in the Au(10)/TRGO nanocomposite. (**h**) STEM/EDS chemical mapping (Au and O; scale bar, 4 nm) of the Au(10)/TRGO hybrid system showing a single gold nanoparticle inside the TRGO matrix.

**Figure 6:** Schematic representation of the approach. A schematic representation of the universal approach for an entrapment of SP nanometals in TRGO matrix starting from a metal-containing molecular precursor and GO. As an example, the scheme depicts the formation of an Fe/TRGO hybrid with ring-like assembly of iron nanoparticles (red) trapped among GO sheets (black). Note: In this schematic representation, the size ratios of individual atoms do not correspond to real conditions. In the structure of iron(III) nitrate, Fe is shown in red, N in yellow and O in blue.

## References

[b1] BatlleX. & LabartaA. Finite-size effects in fine particles: magnetic and transport properties. J. Phys. D: Appl. Phys. 35, R15–R42 (2002).

[b2] NéelL. Théorie du traînage magnétique des ferromagnétiques en grains fins avec applications aux terres cuites. Ann. Geophys. 5, 99–136 (1949).

[b3] BeanC. P. & LivingstonJ. D. Superparamagnetism. J. Appl. Phys. 30, S120–S129 (1959).

[b4] BrownW. F.Jr Relaxation behavior of fine magnetic particles. J. Appl. Phys. 30, S130–S132 (1959).

[b5] DormannJ. L., FioraniD. & TroncE. in *Advances in Chemical Physics* Vol. 98 (eds Prigogine, I. & Rice, S. A.) 283–494 (John Wiley & Sons, 1997).

[b6] BedantaS. & KleemannW. Supermagnetism. J. Phys. D: Appl. Phys 42, 013001 (2009).

[b7] HaiP. N., OhyaS., TanakaM., BarnesS. E. & MaekawaS. Electromotive force and huge magnetoresistance in magnetic tunnel junctions. Nature 458, 489–492 (2009).1927068110.1038/nature07879

[b8] ErbR. M., LibanoriR., RothfuchsN. & StudartA. R. Composites reinforced in three dimensions by using low magnetic fields. Science 335, 199–204 (2012).2224677210.1126/science.1210822

[b9] GeJ. P., HuY. X. & YinY. D. Highly tunable superparamagnetic colloidal photonic crystals. Angew. Chem. Int. Ed. 46, 7428–7431 (2007).10.1002/anie.20070199217610234

[b10] GeJ. P. *et al.* Magnetochromatic microspheres: rotating photonic crystals. J. Am. Chem. Soc. 131, 15687–15694 (2009).1952704910.1021/ja903626h

[b11] ThomasL. *et al.* Macroscopic quantum tunnelling of magnetization in a single crystal of nanomagnets. Nature 383, 145–147 (1996).

[b12] ReddyL. H., AriasJ. L., NicolasJ. & CouvreurP. Magnetic nanoparticles: design and characterization, toxicity and biocompatibility, pharmaceutical and biomedical applications. Chem. Rev. 112, 5818–5878 (2012).2304350810.1021/cr300068p

[b13] LaurentS. *et al.* Magnetic iron oxide nanoparticles: synthesis, stabilization, vectorization, physicochemical characterizations, and biological applications. Chem. Rev. 108, 2064–2110 (2008).1854387910.1021/cr068445e

[b14] GuptaA. K. & GuptaM. Synthesis and surface engineering of iron oxide nanoparticles for biomedical applications. Biomaterials 26, 3995–4021 (2005).1562644710.1016/j.biomaterials.2004.10.012

[b15] LuA. H., SalabasE. L. & SchuthF. Magnetic nanoparticles: synthesis, protection, functionalization, and application. Angew. Chem. Int. Ed. 46, 1222–1244 (2007).10.1002/anie.20060286617278160

[b16] GaoJ. H., GuH. W. & XuB. Multifunctional magnetic nanoparticles: design, synthesis, and biomedical applications. Acc. Chem. Res. 42, 1097–1107 (2009).1947633210.1021/ar9000026

[b17] HolaK., MarkovaZ., ZoppellaroG., TucekJ. & ZborilR. Tailored functionalization of iron oxide nanoparticles for MRI, drug delivery, magnetic separation and immobilization of biosubstances. Biotechnol. Adv. 33, 1162–1176 (2015).2568907310.1016/j.biotechadv.2015.02.003

[b18] UlbrichK. *et al.* Targeted drug delivery with polymers and magnetic nanoparticles: covalent and noncovalent approaches, release control, and clinical studies. Chem. Rev. 116, 5338–5431 (2016).2710970110.1021/acs.chemrev.5b00589

[b19] RanberS. Unexpected magnetism in nanomaterials. J. Magn. Magn. Mater. 346, 58–73 (2013).

[b20] Leslie PeleckyD. L. & RiekeR. D. Magnetic properties of nanostructured materials. Chem. Mater. 8, 1770–1783 (1996).

[b21] SkumryevV. *et al.* Beating the superparamagnetic limit with exchange bias. Nature 423, 850–853 (2003).1281542610.1038/nature01687

[b22] DreyerD. R., ParkS., BielawskiC. W. & RuoffR. S. The chemistry of graphene oxide. Chem. Soc. Rev. 39, 228–240 (2010).2002385010.1039/b917103g

[b23] ZhuY. W. *et al.* Graphene and graphene oxide: synthesis, properties, and applications. Adv. Mater. 22, 3906–3924 (2010).2070698310.1002/adma.201001068

[b24] GeorgakilasV. *et al.* Functionalization of graphene: covalent and non-covalent approaches, derivatives and applications. Chem. Rev. 112, 6156–6214 (2012).2300963410.1021/cr3000412

[b25] YooJ. M., KangJ. H. & HongB. H. Graphene-based nanomaterials for versatile imaging studies. Chem. Soc. Rev. 44, 4835–4852 (2015).2577753010.1039/c5cs00072f

[b26] YangK. *et al.* Graphene in mice: ultrahigh *in vivo* tumor uptake and efficient photothermal therapy. Nano Lett. 10, 3318–3323 (2010).2068452810.1021/nl100996u

[b27] ZhangL. M., XiaJ. G., ZhaoQ. H., LiuL. W. & ZhangZ. J. Functional graphene oxide as a nanocarrier for controlled loading and targeted delivery of mixed anticancer drugs. Small 6, 537–544 (2010).2003393010.1002/smll.200901680

[b28] YangX. Y. *et al.* High-efficiency loading and controlled release of doxorubicin hydrochloride on graphene oxide. J. Phys. Chem. C 112, 17554–17558 (2008).

[b29] YangK., FengL. Z., ShiX. Z. & LiuZ. Nano-graphene in biomedicine: theranostic applications. Chem. Soc. Rev. 42, 530–547 (2013).2305965510.1039/c2cs35342c

[b30] TucekJ., KempK. C., KimK. S. & ZborilR. Iron-oxide-supported nanocarbon in lithium-ion batteries, medical, catalytic, and environmental applications. ACS Nano 8, 7571–7612 (2014).2500053410.1021/nn501836x

[b31] UthaisarC., BaroneV. & FahlmanB. D. On the chemical nature of thermally reduced graphene oxide and its electrochemical Li intake capacity. Carbon 61, 558–567 (2013).

[b32] ShavelA., Rodriguez-GonzalezB., SpasovaM., FarleM. & Liz-MarzanL. M. Synthesis and characterization of iron/iron oxide core/shell nanotubes. Adv. Funct. Mater. 17, 3870–3876 (2007).

[b33] FerrariA. C. *et al.* Raman spectrum of graphene and graphene layers. Phys. Rev. Lett. 97, 187401 (2006).1715557310.1103/PhysRevLett.97.187401

[b34] ChourpaI. *et al.* Molecular composition of iron oxide nanoparticles, precursors for magnetic drug targeting, as characterized by confocal Raman microspectroscopy. Analyst 130, 1395–1403 (2012).1617266510.1039/b419004a

[b35] BodkerF., MorupS. & LinderothS. Surface effects in metallic iron nanoparticles. Phys. Rev. Lett. 72, 282–285 (1994).1005610510.1103/PhysRevLett.72.282

[b36] MargeatO., RespaudM., AmiensC., LecanteP. & ChaudretB. Ultrafine metallic Fe nanoparticles: synthesis, structure and magnetism. Beilstein J. Nanotechnol. 1, 108–118 (2010).2197740010.3762/bjnano.1.13PMC3045918

[b37] LacroixL. M. *et al.* Ultrasmall iron nanoparticles: effect of size reduction on anisotropy and magnetization. J. Appl. Phys. 103, 07D521 (2008).

[b38] MachalaL., ZborilR. & GedankenA. Amorphous iron(III) oxide—a review. J. Phys. Chem. B 111, 4003–4018 (2007).1740277210.1021/jp064992s

[b39] MachalaL., TucekJ. & ZborilR. Polymorphous transformations of nanometric iron(III) oxide: a review. Chem. Mater. 23, 3255–3272 (2011).

[b40] BalettoF. & FerrandoR. Structural properties of nanoclusters: energetic, thermodynamic, and kinetic effects. Rev. Modern Phys. 77, 371–423 (2005).

[b41] KnickelbeinM. B. Magnetic moments of bare and benzene-capped cobalt clusters. J. Chem. Phys. 125, 044308 (2006).10.1063/1.221795116942143

[b42] RohrerM., BauerH., MintorovitchJ., RequardtM. & WeinmannH. J. Comparison of magnetic properties of MRI contrast media solutions at different magnetic field strengths. Invest. Radiol. 40, 715–724 (2005).1623090410.1097/01.rli.0000184756.66360.d3

[b43] NaH. B., SongI. C. & HyeonT. Inorganic nanoparticles for MRI contrast agents. Adv. Mater. 21, 2133–2148 (2009).

[b44] LeeJ. H. *et al.* Artificially engineered magnetic nanoparticles for ultra-sensitive molecular imaging. Nat. Med. 13, 95–99 (2007).1718707310.1038/nm1467

[b45] SeoW. S. *et al.* FeCo/graphitic-shell nanocrystals as advanced magnetic-resonance-imaging and near-infrared agents. Nat. Mater. 6, 971–976 (2006).1711502510.1038/nmat1775

[b46] ProchazkaR. *et al.* Statistical analysis and digital processing of the Mössbauer spectra. Meas. Sci. Technol. 21, 025107 (2010).

